# USP21 Promotes the Progression of Nasopharyngeal Carcinoma by Regulating FOXM1

**DOI:** 10.1155/2023/9196583

**Published:** 2023-02-11

**Authors:** Xiaofeng Li, Xia Li

**Affiliations:** ^1^Department of Otorhinolaryngology, Head and Neck Surgery, Shanghai Jiao Tong University Affiliated Sixth People's Hospital, Shanghai 201306, China; ^2^Department of Otorhinolaryngology, The Second People's Hospital of Changzhou, Changzhou, Jiangsu 213164, China

## Abstract

The purpose of this work was to explore the molecular mechanisms by which USP21 regulates nasopharyngeal carcinoma tumor growth and cancer cell stemness. In this study, the USP21 transcript data was obtained from TCGA database. Then, qPCR and western blot tests revealed that, in contrast to normal tissue or normal nasopharyngeal epithelial cells, the expression of USP21 was greater in nasopharyngeal carcinoma tissues or cell lines, respectively. CCK-8 and EdU immunofluorescent staining assays revealed that USP21 promoted the proliferation of nasopharyngeal carcinoma cells. Meanwhile, scratch and transwell assays showed that USP21 facilitated migration and invasion of nasopharyngeal carcinoma cells. Sphere formation assay was performed on nasopharyngeal carcinoma cells after knockdown of USP21, which revealed that knockdown of USP21 inhibited the stemness profiles of nasopharyngeal carcinoma cells. Then, the western blot assays indicated that knockdown of USP21 in nasopharyngeal carcinoma cells would inhibit FOXM1 expression, and overexpression of FOXM1 could reverse the cell proliferation ability, cell migration and invasion ability, and cell stemness profiles. Finally, a nasopharyngeal xenograft model suggested that USP21 facilitated tumor growth in mice. These findings proved that USP21 promoted tumor growth and cancer cell stemness in nasopharyngeal carcinoma by regulating FOXM1.

## 1. Introduction

In southern China and Southeast Asia, nasopharyngeal carcinoma (NPC) is a common head and neck cancer. Most patients diagnosed with advanced stage III or IV have a poor prognosis and die from local recurrence and metastasis after treatment. However, the underlying mechanism remains largely unknown. Cancer stem cells (CSC) are defined as subpopulations of cells within tumors that have the capacity to self-renew and produce new tumors and are responsible for the infinite proliferation, invasion, and advanced stage of cancer in patients.

The Forkhead box (FOX) family of proteins plays an important role in regulating a wide range of transcriptional activities from cell homeostasis to development. FOXM1 is a protooncogene transcription factor that contributes greatly to cell cycle progression. Endogenous FOXM1 expression regulates the expression of multiple G2/M-specific genes. Conversely, inhibition of FOXM1 leads to reduced proliferation, migration, and metastasis of cancer cells, and FOXM1 is strongly correlated with clinicopathological features of stem cell-related in NPC tissues, such as late clinical stage, tumor recurrence, and distant metastasis. In addition, FoxM1 is highly correlated with the expression levels of Nanog, Sox2, OCT4, and other stem cell markers in tumor samples and can also promote the expression of these stem cell-related genes in vitro. In addition, By expanding side group (SP) cells and growing tumor spheres, FOXM1 also gives cancer cells the ability to self-renew [1].

The ubiquitin-specific protease 21 (USP21), a member of the deubiquitylase (DUB) family, has been noted to play a carcinogenic function in many tumors and can promote non-small-cell lung carcinoma growth, migration, and invasion [2]. USP21 stabilizes MEK2 and promotes tumor growth by reducing polyubiquitination at Lys48 [3]. Inhibition of EZH2 ubiquitination in bladder cancer promotes cell proliferation and metastasis [4]. USP21 deubiquitinates and stabilizes TCF/LEF transcription factor TCF7, thereby promoting pancreatic cancer cell dryness [5]. USP21 binds and deubiquitinates FOXM1 *in vivo* and *in vitro*, thus increasing FOXM1 stability. USP21 depletion makes basal-like breast carcinoma cell lines and mouse xenograft tumors sensitive to paclitaxel [6].

TCGA shows that USP21 is highly expressed in head and neck cancer, but there are few studies investigating on the role of USP21 in nasopharyngeal cancer, and the relevant mechanisms are still unclear. Therefore, this work explored the role of USP21 in regulating nasopharyngeal cancer and the underlying mechanism.

## 2. Materials and Methods

### 2.1. Data Acquisition

The Cancer Genome Atlas (TCGA) database (http://tcga-data.nci.nih.gov) can be used to mine gene databases and analyze the expression profiles of various malignant tumors worldwide including head-neck squamous cell carcinoma (HNSC). The USP21 expression data was obtained from TCGA database for HNSC, including 520 tumor samples and 44 normal samples.

### 2.2. Tissue Sample

Thirty instances of NPC tissue and paracarcinoma tissue samples were obtained from the Second People's Hospital Changzhou from NPC patients. All the patients providing samples were informed and signed informed consents, and they did not receive radiotherapy or chemotherapy prior to sample collection. Research protocols were approved by the Ethics Committee of the Second People's Hospital Changzhou according to the principles established in the Declaration of Helsinki [7] (Approval No. [2017]KY308-01). Clinical information in this study is listed in Table 1.

### 2.3. qPCR

Trizol reagent (Invitrogen) was used to collect total RNA from tissue samples or cells. A NanoDrop 1000 spectrophotometer (Thermo Scientific) was applied to evaluate the integrity and quantity of RNA. SYBR Premix EX Taq™ II (Perfect Real Time, Takara, Japan) was applied to detect the expression of USP21. The PCR reaction was performed by CFX96 Touch Real-Time PCR Detection System (Bio-Rad, USA). The reaction conditions were 10 min of predenaturation at 92°C, 40 cycles of 10 sec at 92°C, and 60 sec at 60°C. Primer sequences are listed in Table 2.

### 2.4. Western Blot

Cells or tissue samples were washed by PBS for four times. Then, the protein was separated by RIPA (Thermo Scientific), electrophoresed to SDS-PAGE, and transferred onto PVDF membranes. After, protein was identified by specific primary antibodies USP21 (ab38864, 1 : 1000; Abcam), Oct4 (ab19857, 1 : 2500; Abcam), Nanog (ab21624, 1 : 3000; Abcam), Sox2 (ab97959, 1 : 2500; Abcam), FOXM1 (ab207298, 1 : 1500; Abcam), and GAPDH (ab9485, 1 : 3000; Abcam) overnight at 4°C. Then, HRP-conjugated goat anti-rabbit IgG secondary antibody (ab205718, 1 : 2000; Abcam) was applied to the membranes, and the bands were visualized by ECL chemiluminescence reagent (Thermo Scientific). The gray level of each band was quantitatively analyzed by ImageJ software.

### 2.5. Cell Culture

Three NPC cell lines (C666-1, SUNE-1, and 5-8F) and the normal human nasopharyngeal epithelial cell line (NP69) were purchased from the Chinese Academy of Sciences. The cells were cultured in DMEM (Gibco, CA, USA) supplemented with 12% FBS (Gibco), and 1% p/s (Gibco) in an incubator with 5% CO_2_.

### 2.6. Cell Transfection

Two different types of shRNA (short hairpin RNA) oligonucleotide sequences that target USP21 as well as a scrambled shRNA as a negative control were also cloned into a vector for USP21 knockdown. In order to confirm the impact of FOXM1 overexpression, cells were transfected with or without vectors containing FOXM1 sequences. GenePharma provided the synthetic sh-USP21#1, sh-USP21#2, sh-NC, pcDNA, and pcDNA-FOXM1 molecules (Shanghai, China). In order to transfect the vectors, Lipofectamine 3000 was used (Invitrogen).

### 2.7. CCK-8 Cell Viability Assay

Using the CCK-8 test, the level of cell viability was determined. 2.5 × 10^3^ transfected cells were plated in duplicate onto 96-well plates, 10 *μ*L of CCK-8 solution (Beyotime) was then added, and cells were then incubated for an additional 4 h. Each sample's optical density value at 450 nm was assessed using a microplate reader (BioTek, Winooski, VT, USA).

### 2.8. EdU (5-Ethynyl-2′-deoxyuridine) Analysis

Briefly, cell proliferation was detected using an EdU kit (Beyotime) according to the protocol and followed by staining with DAPI. Cells doubly stained by EdU and DAPI were considered positive proliferators.

### 2.9. Transwell Assay

For cell invasion assay, cells were plated into transwell inserts (Costar, Manassas, VA, USA) with 210 *μ*L of serum-free medium. For cell migration assay, transwell inserts were precoated with Matrigel (Corning, USA) and cells were plated into transwell inserts with 210 *μ*L of serum-free medium. Thereafter, 590 *μ*L of medium with 10% FBS was added to the well, and cells were continued to grow in the incubator for one day. Then, cells were fixed by 4% paraformaldehyde for 20 minutes and dyed by 0.1% crystal violet for 23 minutes. Cell number was counted after the culture plate was dried.

### 2.10. Scratch Assay

Briefly, cells were cultured in the plate and the surface of the plate was scratched by a pipette tip. Thereafter, the plate was rinsed for several times to remove cells that had been scraped away. Then, the cells were allowed to continue to grow in the incubator, and photos were taken one day after the incubation.

### 2.11. Sphere Formation Assay

N2 and B27 (0.5x, Invitrogen, USA), bFGF and EGF (50 ng/mL, Sino Biological, China), and glutamine (1x, Invitrogen, USA) were added to cells (4.5 × 10^3^ cells/mL) that were cultivated on ultralow adhesion plates in a serum-free media for one week. The tumor spheres that had a diameter greater than 60 *μ*m were then counted.

### 2.12. Animals and Establishment of a Nasopharyngeal Xenograft Model

Vital River Co. Ltd. (Beijing, China) provided male BALB/c nude mice that were 8 weeks old and weighed 17–21 g. All experimental methods were carried out in compliance with the National Institutes of Health Laboratory Animal Care and Use Guidelines after this study was authorized by the animal ethics committee of the Second People's Hospital Changzhou. A mouse's right flank was injected with 2.2 x 10^6^ transfected C666-1 cells, suspended in 210 *μ*L of serum-free media (*n* = 5). Mice were sacrificed after 31 days, and tumor weights and volumes were assessed (Approval No. [2017]KY308-01).

### 2.13. Immunohistochemistry Analysis

Briefly, tissues were first deparaffinized and rehydrated. Then, 0.01 M citrate buffer was used for antigen retrieval. Thereafter, 0.3% hydrogen peroxide was used for 12 minutes to suppress endogenous peroxidase activity. Tissues were then blocked using goat serum and incubated with primary antibodies USP21, FOXM1, and Ki-67 (ab15580, 1 : 3500, Abcam) at 4°C for a whole night. Finally, tissues were treated with fluorescent dye-conjugated secondary antibody (Beyotime) for 1.5 h.

### 2.14. Statistical Analysis

All data was expressed as mean ± standard error of the mean from 3 (except for TCGA, qPCR, and xenograft model) or 5 (xenograft model) independent experiments. Differences between two groups were compared through the Student *t*-test, and differences among multiple groups were compared through one-way analysis of variance (ANOVA). *p* values of <0.01 (two-tailed) were considered statistically significant difference.

## 3. Results

### 3.1. Knockdown of USP21 Inhibited Proliferation of Nasopharyngeal Carcinoma Cells

To investigate the correlation between USP21 expression and nasopharyngeal carcinoma, the clinical data of nasopharyngeal carcinoma expression profile data was obtained from TCGA database. The result revealed that the USP21 transcript was highly expressed in HNSC (*n* = 520) compared to the normal group (*n* = 44) (Figure 1(a)). Then, qPCR and western blot were performed on tumor tissues and adjacent tissues of nasopharyngeal carcinoma patients during surgery to detect USP21 expression levels in this study. Both qPCR (*n* = 30) and western blot (*n* = 3) assays indicated that the protein expression of USP21 was obviously enhanced in tumor tissues (Figures 1(b) and 1(c)). Further, the protein expression of USP21 in human normal human nasopharyngeal epithelial cell line (NP69) and three nasopharyngeal carcinoma cell lines (C666-1, SUNE-1, and 5-8F) was also determined by western blot, respectively. The result indicated that the protein expression of USP21 was significantly increased in all three kinds of nasopharyngeal carcinoma cell lines (Figure 1(d)). To investigate the effects of USP21 on nasopharyngeal carcinoma cell proliferation, two kinds of nasopharyngeal carcinoma cells (C666-1 and 5-8F) were transfected with shRNA control (sh-NC) and two kinds of USP21-targeting shRNA (sh-USP21#1 and sh-USP21#2) to ensure long-term transfection efficiency, respectively. After transfection, the mRNA expression of USP21 in C666-1 and 5-8F was examined. Cells transfected with USP21-targeting shRNA showed markedly lower USP21 expression at the mRNA levels compared to the sh-NC group, which confirmed transfection efficiency (Figure 1(e)). Then, CCK-8 and EdU immunofluorescent staining assays were used to investigate the effect of USP21 on the nasopharyngeal carcinoma cell proliferation. Both CCK-8 and EdU immunofluorescent staining assays indicated that compared with the control group, suppression of USP21 notably inhibited nasopharyngeal carcinoma cell proliferation (Figures 1(f) and 1(g)). These results hinted that USP21 was significantly expressed in nasopharyngeal carcinoma tissues and cell lines, and knockdown of USP21 inhibited proliferation of nasopharyngeal carcinoma cells.

### 3.2. Knockdown of USP21 inhibited the Migration and Invasion of Nasopharyngeal Carcinoma Cells

To examine the effects of USP21 on nasopharyngeal carcinoma cell migration and invasion, transwell and scratch assays were carried out on the above two nasopharyngeal carcinoma cell lines. The transwell assay results hinted that the rate of invaded nasopharyngeal carcinoma cells was dramatically decreased after sh-USP21#1 and sh-USP21#2 transfection (Figure 2(a)). The scratch results proved that the mobility of nasopharyngeal carcinoma cells was obviously enhanced after sh-USP21#1 and sh-USP21#2 transfection (Figure 2(b)). These results proved that knockdown of USP21 inhibited the migration and invasion of nasopharyngeal carcinoma cells.

### 3.3. Knockdown of USP21 Inhibited the Stemness Profiles of Nasopharyngeal Carcinoma Cells

Furthermore, to investigate the effects of USP21 on nasopharyngeal carcinoma cell stemness profiles, *in vitro* sphere formation and western blot assays were performed on above two nasopharyngeal carcinoma cell lines. The *in vitro* sphere formation assay results revealed that knockdown of USP21 obviously reduced the cellular sphere formation capacity of nasopharyngeal carcinoma cells (Figure 3(a)). The number and the average diameter of cellular sphere formation were significantly decreased after sh-USP21#1 and sh-USP21#2 transfection. The western blot assay results showed that knockdown of USP21 negatively regulated the expression of cell stemness-related proteins, such as Oct4, Nanog, and Sox2 (Figure 3(b)). These results suggested that knockdown of USP21 inhibited the stemness profiles of nasopharyngeal carcinoma cells.

### 3.4. USP21 Promoted Nasopharyngeal Carcinoma Progression through FOXM1

To estimate the mechanism of USP21 promoting the migration, invasion, and stemness profiles of nasopharyngeal carcinoma cells by the FOXM1 pathway, western blot assay was used to check the expression of FOXM1 in nasopharyngeal carcinoma cells after sh-USP21#1 and sh-USP21#2 transfection. The western blot assay results indicated that USP21 positively regulated FOXM1 expression (Figure 4(a)). Furthermore, C666-1 was transfected with sh-USP21#1 and pcDNA/pcDNA-FOXM1, respectively. After transfection, the mRNA expression of FOXM1 in C666-1 was examined. Cells transfected with FOXM1 overexpression vector showed dramatically higher FOXM1 expression at the mRNA levels, which confirmed transfection efficiency (Figure 4(b)). Then, CCK-8 assay was used to check the effect of FOXM1 on nasopharyngeal carcinoma cell proliferation. The CCK-8 assay indicated that compared with the control group, suppression of USP21 notably inhibited nasopharyngeal carcinoma cell proliferation ability, while overexpression of FOXM1 obviously reversed the cell proliferation ability of nasopharyngeal carcinoma cell lines (Figure 4(c)). Meanwhile, the transwell assay results hinted that the rate of invaded nasopharyngeal carcinoma cells was dramatically decreased after knocking down USP21, while overexpression of FOXM1 dramatically reversed the cell migration and invasion ability of nasopharyngeal carcinoma cell lines (Figure 4(d)). Besides, the *in vitro* sphere formation assay results revealed that knockdown of USP21 obviously reduced the cellular sphere formation capacity of nasopharyngeal carcinoma cells, while overexpression of FOXM1 strikingly reversed the cell stemness profiles of nasopharyngeal carcinoma cells (Figure 4(e)). These results proved that USP21 promoted nasopharyngeal carcinoma progression through regulating FOXM1 expression.

### 3.5. Knockdown of USP21 Inhibited Tumor Growth *In Vivo*

Ultimately, to check the effects of USP21 on nasopharyngeal carcinoma *in vivo*, C666-1 transfected with sh-USP21#1 were injected into the mouse to induce tumor formation. The nasopharyngeal xenograft model confirmed that the tumor volume and weight of mice injected with sh-USP21#1-transfected cells were smaller and lower than those of mice injected with sh-NC-transfected cells, indicating that knockdown of USP21 can inhibit tumor growth *in vivo* and USP21 can promote tumor growth in mice (Figure 5(a)). The protein expression level of USP21, FOXM1, and Ki-67 in nasopharyngeal carcinoma tumors in mice was examined. Cells transfected with sh-USP21#1 showed markedly lower USP21, FOXM1, and Ki-67 protein expression, which confirmed transfection efficiency and showed that USP21 promoted tumorigenesis *in vivo* through FOXM1 (Figure 5(b)).

## 4. Discussion

NPC is a kind of epithelial cancer commonly found in the nasopharyngeal crypt. Data from the International Agency for Research on Cancer (IARC) shows that the number of new cases of NPC in 2020 is close to 200,000, and the geographical distribution of NPC in the world is unbalanced [8]. Genetic, ethnic, and environmental factors are all influential factors for the incidence of NPC. NPC is often treated with radiotherapy, and the large differences in tumor biology between patients lead to poor prognoses. NPC with malignant degree is higher, highly aggressive, and prone to local infiltration and neck lymph node metastasis; a lot of patients with nasopharyngeal carcinoma are not diagnosed until late, so the survival rate is low [9, 10]. How to effectively predict the invasion and metastasis of NPC potential, looking for potential molecular therapeutic targets, to select the appropriate treatment plan and prognosis is of great significance. In the present study, the results addressed that USP21 transcript was highly expressed in nasopharyngeal carcinoma compared to the normal group. The protein expression of USP21 was also obviously enhanced in tumor tissues and nasopharyngeal carcinoma cell lines.

USP21 is a ubiquitin-specific hydrolase in the USP family, which plays an important role in regulating cell signal transduction and disease development [11]. USP21 is a cytoplasmic shuttle protein, whose N-terminal nuclear output signal sequence can bind to and mediate the exportation of nuclear output receptor, thus regulating its localization and deubiquitination of its highly conserved cysteine and histidine domains [12]. In recent years, it has been found that USP21 regulates the progression of different tumors. In our study, the result showed that suppression of USP21 notably inhibited nasopharyngeal carcinoma cell proliferation, migration, invasion, and cellular sphere formation ability. Furthermore, the nasopharyngeal xenograft mouse model also suggested that USP21 facilitated tumor growth in mice. However, further morphological analysis of human tissue samples should be carried out in subsequent experiments.

Oct4, Nanog, and Sox2 play a synergistic role in regulating cell stemness profiles, and it has been confirmed that the central “headquarters” composed of Oct4, Nanog, and Sox2 maintain the continuous self-renewal ability and high differentiation potential of cells in the undifferentiated state [13]. The Oct4/Nanog/Sox2 complex is formed by the binding of Nanog and Sox2 to the CR4 and CR2 regions of Oct4. The heterodimer complex formed by Oct4/Sox2 can activate the transcriptional activity of Oct4 itself and further activate the signaling pathway to maintain cell stemness profiles [14]. In our study, the result confirmed that knockdown of USP21 negatively regulated the expression levels of cell stemness-related proteins, such as Oct4, Nanog, and Sox2, suggesting that knockdown of USP21 inhibited the stemness profiles of nasopharyngeal carcinoma cells.

FOXM1 is a member of the Forkhead transcription factor family, which is a family of proteins with a helix DNA domain [15]. FOXM1 is reported to be highly expressed in basal cell carcinoma, hepatocellular carcinoma, lung cancer, and breast cancer cells and can regulate the cell growth cycle and promote the proliferation and differentiation of tumor cells [16]. In our study, the results showed that USP21 positively regulated FOXM1 expression, and overexpression of FOXM1 could reverse the cell proliferation ability, cell migration and invasion ability, and cell stemness profiles, suggesting that USP21 promoted nasopharyngeal carcinoma progression through regulating FOXM1 expression.

In conclusion, this study demonstrated the mRNA and protein expression of USP21 was higher in nasopharyngeal carcinoma tissues or cell lines than normal tissue or normal nasopharyngeal epithelial cells, respectively. In addition, downregulation of USP21 inhibited proliferation, migration, invasion, and stemness profiles of nasopharyngeal carcinoma cells. Further research indicated that USP21 promoted nasopharyngeal carcinoma progression through regulating FOXM1 expression. Meanwhile, the nasopharyngeal xenograft model was established to verify if knockdown of USP21 inhibited tumor growth *in vivo*. Therefore, our results indicated that USP21 promoted tumor growth and cancer cell stemness in nasopharyngeal carcinoma by regulating FOXM1 expression, which could pave the way for advanced therapeutic targets for NPC.

## Figures and Tables

**Figure 1:** Knockdown of USP21 inhibited proliferation of nasopharyngeal carcinoma cells. (a) The USP21 transcript clinical data of nasopharyngeal carcinoma expression profile data in TCGA database. (b, c) The mRNA and protein expression levels of USP21 in tumor tissues and adjacent tissues of nasopharyngeal carcinoma patients. (d) The protein expression levels of USP21 in human normal human nasopharyngeal epithelial cell line (NP69) and three nasopharyngeal carcinoma cell lines (C666-1, SUNE-1, and 5-8F). (e) Knockdown of USP21 in C666-1 and 5-8F nasopharyngeal carcinoma cell lines was verified by western blot. (f, g) Serial CCK-8 and EdU cell viability assays were used to detect the proliferation of C666-1 and 5-8F nasopharyngeal carcinoma cell lines after knocking down USP21. Data was presented as the mean ± SD with three independent experiments. ^∗∗^*p* < 0.01 and ^∗∗∗^*p* < 0.001 versus the control group.

**Figure 2:** Knockdown of USP21 inhibited the migration and invasion of nasopharyngeal carcinoma cells. (a) Transwell assay of C666-1 and 5-8F nasopharyngeal carcinoma cell lines with knockdown of USP21. (b) Wound scratch healing assay of C666-1 and 5-8F nasopharyngeal carcinoma cell lines with knockdown of USP21. Data was presented as the mean ± SD with three independent experiments. ^∗^*p* < 0.05, ^∗∗^*p* < 0.01, and ^∗∗∗^*p* < 0.001 versus the control group.

**Figure 3:** Knockdown of USP21 inhibited the stemness profiles of nasopharyngeal carcinoma cells. (a) Sphere formation assays of C666-1 and 5-8F nasopharyngeal carcinoma cell lines with knockdown of USP21. (b) The protein expression levels of cell stemness-related proteins in C666-1 and 5-8F nasopharyngeal carcinoma cell lines with knockdown of USP21. ^∗^*p* < 0.05, ^∗∗^*p* < 0.01, and ^∗∗∗^*p* < 0.001 versus the control group.

**Figure 4:** USP21 promoted nasopharyngeal carcinoma progression through FOXM1. (a) The protein expression levels of FOXM1 in C666-1 nasopharyngeal carcinoma cell line with knockdown of USP21. (b) The protein expression levels of FOXM1 in C666-1 nasopharyngeal carcinoma cell line with knockdown of USP21 and overexpression of FOXM1. (c) Serial CCK-8 cell viability assay detected the proliferation of the C666-1 nasopharyngeal carcinoma cell line with knockdown of USP21 and overexpression of FOXM1. (d) Transwell assay of the C666-1 nasopharyngeal carcinoma cell line with knockdown of USP21 and overexpression of FOXM1. (e) Sphere formation assays of the C666-1 nasopharyngeal carcinoma cell line with knockdown of USP21 and overexpression of FOXM1. ^∗∗^*p* < 0.01 and ^∗∗∗^*p* < 0.001 versus the control group, ^##^*p* < 0.01 and ^###^*p* < 0.001 versus knockdown of the USP21 group.

**Figure 5:** Knockdown of USP21 inhibited tumor growth *in vivo*. (a) Tumor volume and weight in mice after transfected cells were injected. (b) The protein expression levels of USP21, FOXM1, and Ki-67 in C666-1 nasopharyngeal carcinoma tumors in mice with knockdown of USP21. Data was presented as the mean ± SD with three independent experiments. ^∗∗∗^*p* < 0.001 versus the control group.

**Table 1:** The relationship between the expression level of USP21 and the clinicopathological characteristics in NPC.

Characteristics	Number of patients	TSPAN1 low expression	TSPAN1 high expression	*p* value
Number	30	15	15	
Ages (years)				0.464
≤60	17	9	8	
>60	13	6	7	
Gender				0.269
Male	17	10	7	
Female	13	5	8	
TNM stage				0.025^∗^
I + II	18	12	6	
III + IV	12	3	9	
Metastasis				0.028^∗^
No	14	10	4	
Yes	16	5	11	
Differentiation				0.273
Undifferentiated	15	9	6	
Low and moderately differentiated	15	6	9	

**Table 2:** Primers for USP21 and reference genes.

Gene	Primer	Sequence(5′→3′)
USP21	Forward	GTATGCCCTTTGCAACCACT
(27005)	Reverse	GGTGCCAGAGCTTAGAGGTG
GAPDH	Forward	GACTCATGACCACAGTCCATGC
(2597)	Reverse	AGAGGCAGGGATGATGTTCTG

## Data Availability

All data generated or analyzed during this study are included in this published article.
